The article "Screening of Risk Factors for Poor Prognosis in Patients with Refractory Epilepsy Secondary to Encephalomalacia" was retracted in 2023. Reasons: signs of a paper mill; compromised peer review; unreliable results or conclusions.

# Screening of Risk Factors for Poor Prognosis in Patients with Refractory Epilepsy Secondary to Encephalomalacia

**DOI:** 10.1155/2022/5720102

**Published:** 2022-07-04

**Authors:** Yinjun Zhong

**Affiliations:** First People's Hospital of Linping District, Hangzhou 311100, China

## Abstract

**Objective:**

The study was aimed at screening the independent prognostic risk factors for refractory epilepsy associated with encephalomalacia (REAE).

**Methods:**

Patients with REAE treated in the First People's Hospital of Linping District from January 2018 to December 2019 were selected. The prognosis was represented by Engel grading. Clinical data of the patients were collected, including age, sex, BMI, lesion sites, number of lesion sites, lesion size, seizure frequency, epilepsy type, and treatment methods. Independent risk factors for poor prognosis were screened by logistic regression analysis. The receiver operating characteristic curve (ROC) was used to evaluate the prognostic efficacy of independent risk factors.

**Results:**

A total of 48 patients were included in this study, including 31 patients (64.58%) in the good prognosis group and 17 patients (35.42%) in the poor prognosis group. The mean age of the poor prognosis group was higher than that of the good prognosis group (*P* = 0.002). The proportion of patients with multisite lesions in the poor prognosis group was higher than that in the good prognosis group (*P* = 0.016). The proportion of patients with cerebral malacia lesion diameter ≥ 3 cm in the poor prognosis group was higher than that in the good prognosis group (*P* = 0.002). The proportion of patients with attack frequency ≥ 2 times/month in the poor prognosis group was higher than in the good prognosis group (*P* = 0.002). The proportion of patients receiving surgical treatment in the poor prognosis group was lower than that in the good prognosis group (*P* < 0.001). Age, number of lesion sites, size of encephalomalacia, and seizure frequency were independent risk factors for the prognosis of patients with REAE (OR > 1, *P* < 0.05). Surgical treatment was an independent protective factor associated with the prognosis of patients with REAE (OR < 1, *P* < 0.05). The area under the ROC curve of surgical treatment was 0.83 (*P* = 0.004). The area under the ROC curve of the size of encephalomalacia was 0.72 (*P* = 0.008). There was a positive correlation between age and size of encephalomalacia and Engel grade (*r* > 0, *P* < 0.05). Surgical treatment was negatively correlated with Engel grade (*r* < 0, *P* < 0.05). The number of lesion sites and seizure frequency had no significant correlation with Engel (*P* > 0.05). The proportion of Engel I patients treated with surgery was higher than that treated with drugs (*P* = 0.001). The ratio of Engel III and IV patients treated with surgery was lower than that treated with medications (*P* < 0.05).

**Conclusion:**

Age, number of lesion sites, size of encephalomalacia, and seizure frequency are independent risk factors for the prognosis of patients with REAE. Surgical treatment is an independent prognostic factor for patients with REAE. Surgical treatment can significantly improve patient outcomes.

## 1. Introduction

Epilepsy is a common central nervous system disease characterized by paroxysmal, characteristic, repetitive, and stereotyped [1]. Epilepsy is a relatively benign disease. Most epilepsy has a good prognosis, completely controlling seizures and eventually stopping relevant drugs [2]. Intractable epilepsy secondary to encephalomalacia is common in clinics. The disease has a unique pathological basis. The scar of brain tissue pulls the surrounding neuronal cells, resulting in abnormal discharge [3]. Patients with this type of epilepsy are not sensitive to drug treatment, the clinical symptoms are prolonged, and the prognosis is relatively poor [3, 4]. Previous studies have shown that the factors affecting the prognosis of intractable epilepsy include etiology, abnormal EEG, epilepsy type, number of seizures before treatment, and early effect of drugs [5–7]. Sensitive to the early response of treatment indicates that the prognosis of patients is good, and a large number of epileptic seizure history and intellectual disabilities suggest that the prognosis of patients is poor. However, the prognosis of epilepsy is dynamic and variable. Appropriate treatment and active prevention strategies for risk factors can significantly improve the prognosis of patients [8]. There is currently a lack of clinical studies to screen for independent risk factors for poor prognosis in epilepsy. Clinicians cannot accurately assess the prognosis of patients with refractory epilepsy secondary to encephalomalacia. For patients, there is a lack of reasonable follow-up strategies and timely medical interventions. In the study, logistic regression analysis was used to screen independent risk factors related to the prognosis of refractory epilepsy secondary to encephalomalacia. The predictive power of independent literature factors on patient prognosis was assessed by receiver operating characteristic curve (ROC). The study also compared the effects of surgical treatment and medical treatment on patient outcomes. Our research provides a reference for assessing patient prognosis and formulating clinical treatment plans and prevention strategies.

## 2. Materials and Methods

### 2.1. Case Selection

Patients with intractable epilepsy secondary to encephalomalacia treated in the First People's Hospital of Linping District from January 2018 to December 2019 were selected. Inclusion criteria were as follows: (1) the patients met the diagnostic criteria for intractable epilepsy in the diagnostic criteria for epilepsy of the international alliance against epilepsy (2014 Edition), (2) the patient has evidence of encephalomalacia foci, (3) the patient's age is between 18 and 75 years old, and (4) patients were fully aware of the study and signed informed consent. Exclusion criteria were as follows: (1) the patient had a history of brain malignant tumor; (2) the patient has other neurological, mental diseases; (3) poor patient compliance; (4) the patient was complicated with organic diseases of essential organs such as heart, liver, and kidney; (5) patients participated in other clinical trials in recent three months. The hospital ethics committee approved this study.

### 2.2. Prognosis Evaluation

All enrolled patients underwent surgical resection of encephalomalacia foci combined with drug therapy or drug therapy alone, according to the patient's condition and willingness. The patients were followed up for a long time to observe the seizure during the follow-up period. According to the examination results, patients without seizures for more than 2 years can decide whether to reduce the drug dose or stop taking drugs. The prognosis was evaluated according to the Engel classification. Engel grade I was considered as a good prognosis, and Engel grades II, III, and IV were considered as poor prognosis.

### 2.3. Clinical Variable Observation

The clinical data of patients were collected, including age, gender, BMI, lesion location, number, size of cerebromalacia, seizure frequency, epilepsy type, and treatment method. All patients underwent cranial MRI and EEG. The examination results showed that all patients had encephalomalacia, and multiple lesions refer to encephalomalacia involving more than 2 lobes. The size of encephalomalacia was obtained from MRI images and the cumulative lesion diameter of patients with multiple lesions. The type of epileptic seizure is determined according to the classification and term definition of epilepsy by the International Antiepilepsy Alliance in 2017. According to the clinical symptoms and EEG results, the types of seizures were divided into focal seizures, generalized seizures, and seizures of unknown origin.

### 2.4. Statistical Analysis

All data in this study were statistically analyzed by SPSS (24.0). The measurement data were expressed in the form of mean ± standard deviation (*x* ± *s*), and *t*-test was used for comparison between groups. The count data were expressed in the form of a number of cases and rate (*n* (%)), and the chi-square test was used for comparison between groups. Independent risk factors for poor prognosis were screened by logistic regression analysis. The receiver operating characteristic curve (ROC) was used to evaluate the predictive efficacy of independent risk factors on the prognosis of patients. The correlation was analyzed by the Spearman test. *P* < 0.05 means statistically significant.

## 3. Results

### 3.1. Comparative Analysis of Clinical Variables between Good Prognosis Group and Poor Prognosis Group

A total of 48 patients were included in this study, including 31 patients in the good prognosis group (64.58%) and 17 patients in the poor prognosis group (35.42%). The average age of the poor prognosis group was higher than that of the good prognosis group (*P* = 0.002). The ratio of patients with multiple lesions in the poor prognosis group was higher than that in the good prognosis group (*P* = 0.016). Patients with cerebral malacia ≥ 3 cm in the poor prognosis group were higher than that in the good prognosis group (*P* = 0.002). The proportion of patients with seizure frequency ≥ 2 times/month in the poor prognosis group was higher than in the good prognosis group (*P* = 0.002). The proportion of patients receiving surgical treatment in the poor prognosis group was lower than that in the good prognosis group (*P* < 0.001). No significant difference was observed between the good prognosis group and the poor prognosis group in gender, BMI, encephalomalacia lesion location, and epilepsy type (*P* > 0.05), as shown in Table 1.

### 3.2. Screening of Independent Risk Factors Related to Prognosis

The patient's prognosis was taken as the dependent variable (good prognosis = 0, poor prognosis = 1), and the number of lesion parts (single site lesion = 0, multisite lesion = 1), seizure frequency (seizure frequency < 2 times/month = 0, seizure frequency > 2 times/month = 1), and treatment mode (drug treatment = 0, surgical treatment = 1) was taken as the categorical independent variables. Age and the size of encephalomalacia were continuous independent variables for logistic regression analysis. Age, the number of lesions, the size of encephalomalacia, and the frequency of seizures were independent risk factors related to the prognosis of patients with intractable epilepsy secondary to encephalomalacia (OR > 1, *P* < 0.05). Surgical treatment was an independent protective factor related to the prognosis of patients with intractable epilepsy secondary to encephalomalacia (OR < 1, *P* < 0.05), as shown in Table 2.

### 3.3. Evaluation of Prognostic Efficacy of Risk Factors

The area under the ROC curve of prognostic independent risk factors and protective factors in patients with intractable epilepsy secondary to encephalomalacia was calculated, as shown in Figures 1–5. The area under the surgical treatment curve was 0.83, and the prediction efficiency was the best (*P* = 0.004). The immunity under the size curve of encephalomalacia was 0.72, followed by the predictive efficacy (*P* = 0.008), as shown in Table 3.

### 3.4. Correlation between Risk Factors and Engel Classification

Correlation analysis showed that age and the size of encephalomalacia were positively correlated with Engel grade (*r* > 0, *P* < 0.05). There was a negative correlation between surgical treatment and Engel (*r* < 0, *P* < 0.05). The number of lesions and seizure frequency were not significantly correlated with Engel (*P* > 0.05), as shown in Table 4.

### 3.5. Comparison of Engel Classification between Surgical and Drug Treated Patients

The proportion of Engel grade I patients treated with surgery was higher than that treated with drugs (*P* = 0.001). The proportion of patients with Engel III and Engel IV treated by surgery was lower than that treated by drug (*P* < 0.05). There was no significant difference between surgical and drug treatment in Engel grade II patients (*P* > 0.05), as shown in Table 5.

## 4. Discussion

A variety of causes can lead to liquefaction and necrosis of brain tissue and the formation of encephalomalacia [9]. These causes include trauma, cerebrovascular disease, and intracranial infection [10]. The pathological manifestations of brain soft focus ranged from early neuronal necrosis to neuronal disappearance and then to glial cell proliferation. There are no nerve cells in the brain softening focus, which does not cause epileptic discharge. The real pathological site of epileptic discharge is the peripheral nerve tissue [11]. The traction of fibrous scar tissue in the brain can embed the remaining normal neurons cause abnormal discharge and disrupt the function of intertwined proliferative cells. It affects the electrical activity of normal neurons, resulting in seizures. A study suggested that glial cells can lead to epileptic seizures through mechanisms such as increasing the excitability of normal neurons, neuronal cluster discharge, and failure to inhibit the excitability of neurons [12].

In this study, Engel grade was used as a prognostic index for patients with epilepsy. Engel classification is a commonly used criterion for evaluating the efficacy of epilepsy, which can accurately characterize the prognosis of patients [13, 14]. In our study, the proportion of patients with epilepsy with a poor prognosis was 35.42%. Previous research results showed that the proportion of patients with epilepsy with a poor prognosis was about 10% [15–17]. There is such a difference, which may be because we only target refractory epilepsy. Drug resistance or insensitivity to early treatment is the influencing factors of poor prognosis in patients with epilepsy [18–21]. One study showed that [5], after treatment, 2% of patients with epilepsy had no seizures. 53.1% of epileptic patients had a good prognosis, and 22.8% of epileptic symptoms improved. 22.1% of patients with epilepsy had a poor prognosis and showed drug resistance. After multivariate analysis, early seizures, multiple seizure types, and history of status epilepticus were predictive variables of adverse reactions in the early stage of treatment. Early treatment response had a significant positive predictive value at the end of follow-up. After long-term follow-up, initial nonresponse to treatment was an independent risk factor for adverse outcomes.

This study found that age, the number of lesions, the size of encephalomalacia, and the frequency of seizures were independent risk factors related to the prognosis of patients with intractable epilepsy secondary to encephalomalacia. Surgical treatment is an independent protective factor associated with the prognosis of patients with intractable epilepsy secondary to encephalomalacia. Surgical treatment is the best predictor of prognosis among these risk factors and protective factors. And surgical treatment can significantly improve the Engel grade of patients. It is consistent with previous research results. In a single-center retrospective study of 383 patients with epilepsy, 11.8% developed permanent epilepsy [22]. The study found that complete resection of the lesion, disappearance of postoperative epileptic activity, localized histological findings, and lower operative age were significantly associated with good seizure outcomes [22]. Surgical treatment of extratemporal epilepsy can achieve satisfactory results [23–25]. Young patients with localized MRI lesions can obtain the best results and are entirely resected [26]. A study showed that surgical treatment has obvious advantages compared with drug treatment, and the proportion of patients without seizures is higher. However, surgical treatment is not ideal when there are multiple lobar lesions, which is inferior to that of single lobar lesions. Seizure-free outcomes were similar in children and adults. Hippocampal sclerosis and benign tumors have a better prognosis than other pathology. It is considered that seizure activity can be reduced compared with the treatment of epilepsy. The study also pointed out that although the effect of surgical treatment is good, patients with intractable epilepsy still rarely receive surgical treatment [27].

There are some limitations in the study. First, the study lacks external cohort validation. External cohorts can provide stronger evidence and make conclusions more convincing. The second is the need to include more prognostic indicators. It should be noted that the prognosis of epilepsy is closely related to the impact of sociological function. Patients' quality of life, psychological depression, and anxiety can be included in the prognostic indicators: family support, psychological counselling, economic conditions, social support, and other social psychological factors can be included in clinical variables.

In conclusion, age, the number of lesions, the size of encephalomalacia, and the frequency of seizures are independent risk factors related to the prognosis of patients with intractable epilepsy secondary to encephalomalacia. Surgical treatment is an independent protective factor associated with the prognosis of patients with intractable epilepsy secondary to encephalomalacia. Surgical treatment can significantly improve the prognosis of patients.

## Figures and Tables

**Figure 1:** The predictive power of age on prognosis in patients with refractory epilepsy secondary to encephalomalacia. AUC: area under the curve; CI: confidence interval.

**Figure 2:** The predictive efficacy of the number of lesions on the prognosis of patients with refractory epilepsy secondary to encephalomalacia. AUC: area under the curve; CI: confidence interval.

**Figure 3:** The predictive efficacy of encephalomalacia size on the prognosis of patients with refractory epilepsy secondary to encephalomalacia. AUC: area under the curve; CI: confidence interval.

**Figure 4:** Efficacy of seizure frequency in predicting prognosis in patients with refractory epilepsy secondary to encephalomalacia. AUC: area under the curve; CI: confidence interval.

**Figure 5:** Prognostic predictive power of surgical treatment in patients with refractory epilepsy secondary to encephalomalacia. AUC: area under the curve; CI: confidence interval.

**Table 1:** Comparative analysis of clinical variables between good prognosis group and poor prognosis group.

	Good prognosis (*n* = 31)	Poor prognosis (*n* = 17)	*t*/*χ*^2^	*P* value
Age	34.78 ± 10.16	48.23 ± 18.34	3.283	0.002
Sex				
Male	18 (58.06)	9 (52.94)	0.117	0.732
Female	13 (41.94)	8 (47.06)		
BMI	24.16 ± 6.17	24.03 ± 5.62	0.072	0.943
Lesion site				
Temporal lobe	16 (39.02)	17 (43.59)	1.855	
Frontal lobe	13 (31.71)	14 (35.90)		
Parietal lobe	4 (12.90)	2 (11.76)		0.757
Insular lobe	6 (19.35)	3 (17.65)		
Other	2 (6.45)	3 (17.65)		
Lesion number				
Multiple site lesions	6 (19.35)	9 (52.94)	5.765	0.016
Single site lesion	25 (80.65)	8 (47.06)		
Size				
Diameter < 3 cm	26 (83.87)	7 (41.18)	9.315	0.002
Diameter ≥ 3 cm	5 (16.13)	10 (58.82)		
Seizure frequency				
< 2 times/month	20 (64.52)	4 (23.53)	7.378	0.007
≥2 times/month	11 (35.48)	13 (76.47)		
Epilepsy type				
Focal attack	23 (74.19)	14 (82.35)	0.414	0.520
Generalized seizure	8 (25.81)	3 (17.65)		
Treatment method				
Surgical treatment	23 (74.19)	3 (17.65)	14.141	<0.001
Medication	8 (25.81)	14 (82.35)		

**Table 2:** Screening of independent risk factors related to prognosis in patients with intractable epilepsy secondary to encephalomalacia.

Variables	OR	95% CI		*P* value
		Upper limit	Lower limit	
Age	1.23	0.83	1.42	0.031
Lesion number	1.36	0.74	2.21	0.004
Size of encephalomalacia	1.41	1.01	1.89	0.019
Seizure frequency	1.15	0.73	1.93	0.028
Surgical treatment	0.46	0.13	0.73	0.002

**Table 3:** Prognostic efficacy of risk factors in patients with intractable epilepsy secondary to encephalomalacia.

Risk factors	AUC	95% CI		*P* value
		Upper limit	Lower limit	
Age	0.61	0.56	0.87	0.014
Lesion number	0.67	0.38	0.73	0.029
Size of encephalomalacia	0.72	0.35	0.81	0.008
Seizure frequency	0.53	0.41	0.88	0.073
Surgical treatment	0.83	0.62	0.96	0.004

**Table 4:** Correlation between risk factors and Engel classification.

Risk factors	*r*	95% CI		*P* value
		Upper limit	Lower limit	
Age	0.23	0.14	0.77	0.044
Lesion number	0.21	0.15	0.85	0.219
Size of encephalomalacia	0.32	0.26	1.00	0.038
Seizure frequency	0.18	-0.07	0.69	0.361
Surgical treatment	-0.38	-0.64	0.25	0.017

**Table 5:** Comparison of Engel classification between surgical and drug treated patients.

Engel	Surgical-treated (*n* = 26, %)	Medicine-treated (*n* = 22, %)	*χ* ^2^	*P* value
I	22 (84.62)	5 (22.73)	22.501	<0.001
II	2 (23.08)	3 (13.64)	0.451	0.502
III	1 (3.85)	8 (36.36)	8.271	0.004
IV	1 (3.85)	6 (27.27)	5.250	0.022

## Data Availability

The labeled dataset used to support the findings of this study are available from the corresponding author upon request.
